# Analysis of the Characteristics of Dominant Diseases in Traditional Chinese Medicine: Based on 95 Diseases

**DOI:** 10.1155/2022/6972663

**Published:** 2022-06-06

**Authors:** Hanting Wu, Yi Liang, Qiushuang Li, Peijie Hei, Juan Liang, Rongchen Dai, Conghua Ji

**Affiliations:** ^1^School of Public Health, Zhejiang Chinese Medical University, Hangzhou, China; ^2^The Third Affiliated Hospital of Zhejiang Chinese Medical University, Hangzhou, China; ^3^The First Affiliated Hospital of Zhejiang Chinese Medical University, Hangzhou, China

## Abstract

**Background:**

Traditional Chinese medicine (TCM) has been widely used all over the world and has shown its superiority in some diseases. However, there are no clear evaluation criteria for TCM. In 2019, a list of TCM dominant diseases was published by the Chinese National Administration of Traditional Chinese Medicine. This study aimed to systematically summarize the characteristics of 95 TCM dominant diseases and provide a reference for the establishment of evaluation criteria for TCM dominant diseases.

**Methods:**

The diagnosis and treatment protocols of all the 95 TCM dominant diseases were screened. The data of disease classification, diseases' code of TCM, length of hospital stay, treatment protocols, and clinical pathways were reviewed and summarized.

**Results:**

The diseases of the genitourinary and nervous systems accounted for 14.74% and 12.73% of the TCM dominant diseases, respectively. The length of hospital stay for 55 (57.89%) diseases was no more than less than 14 days. Each disease had its specific Chinese herbal decoction pieces and Chinese patent drugs. Chinese medical injections were not widely used. TCM external treatments for these diseases are abundant, with hundreds optional.

**Conclusion:**

Some potentially promising TCM dominant diseases remain to be identified and deserve further research to establish the evaluation criteria of TCM dominant diseases.

## 1. Introduction

TCM has been widely used in the treatment of various diseases in China for thousands of years and has shown its potential and superiority in many diseases such as leukemia, irritable bowel syndrome, and angina pectoris [1–5]. Therefore, the conception of TCM dominant diseases was born. The dominant diseases of TCM mainly refer to diseases for which there is currently no targeted western medical treatment and TCM has a definite effect, or the toxic side effects and drug-induced, iatrogenic disorders of TCM were less than western therapy [6]. For example, some chronic respiratory diseases, such as asthma and chronic obstructive pulmonary disease (COPD), are commonly treated with corticosteroids, which are often accompanied by side effects [7]. Based on conventional therapies, the application of TCM not only significantly improved the symptom of acute exacerbations of COPD (AECOPD) but also reduced hospital stay (mean difference, −1.21 days; *P*=0.003) and the number of AECOPD readmissions (RR, 0.41; *P*=0.015), greatly reducing the overall burden of disease [8].

The evaluation criteria of dominant diseases of TCM are used to define a certain disease as the dominant disease of TCM. However, the criteria should be recognized by the majority of medical workers before it is beneficial for better clinical promotion and application of TCM to provide patients with better curative medical services. Currently, the consensus within countries or industries concerning the evaluation criteria and evaluation tools for dominant diseases of TCM has not been reached yet [9]. There are no mature evaluation systems for the definition of TCM's dominant diseases.

Commissioned by the Chinese National Administration of Traditional Chinese Medicine, the China Association of Chinese Medicine assembled a panel of TCM experts from across the country in 2018 to systematically collect and summarize opinions on dominant diseases of TCM. In 2019, a list of 95 dominant diseases of TCM was published by the Chinese National Administration of Traditional Chinese Medicine with the diagnosis, treatment program, and clinical pathway of these diseases [10]. Definite Chinese medical treatment options, clinical pathway, and objective evaluation criteria of the clinical efficacy were established for these diseases through clinical practice, with broad consensus. This study was conducted to comprehensively summarize the classification of these TCM dominant diseases and the application of TCM treatment, aiming to identify the characteristics of the 95 dominant diseases of TCM and provide a reference for the further selection of TCM dominant diseases and establishment of clear evaluation criteria.

## 2. Methods

### 2.1. Data Sources

The 95 TCM dominant diseases, promulgated by the Chinese National Administration of Traditional Chinese Medicine, were selected as the subjects of this study. Basic information about the International Classification of Diseases (ICD) 10 code [11], ICD 11-code [12], disease classification, and length of hospital stay was collected. Chinese medical treatment protocols were categorized as TCM (oral TCM decoction, oral Chinese patent medicine, and TCM injection) and external treatment of TCM (including external treatment of TCM, acupuncture, moxibustion, manipulation, anorectal of TCM, special therapy of TCM, and comprehensive therapy of TCM).

ICD is a health statistics coding tool and is widely used in clinical practice. Based on ICD 10, substantial improvement was made in ICD 11. More unique codes for injuries and diseases and a new chapter focusing on traditional medicine were also included in ICD 11 [12].

### 2.2. Data Extraction

The diagnosis and treatment protocols of each disease were screened and data were extracted by two researchers independently using a standard data extraction table. Then, they crosschecked the table after primary extraction. Disagreements were resolved through discussion or the suggestion of a third reviewer. The main contents of the table were as follows: disease, classification of diseases, diseases' code of TCM, length of hospital stay, diseases' name in western medicine, code in ICD-10 and ICD-11, optional TCM therapies, and optional TCM external therapies.

### 2.3. Statistical Methods

Statistical analyses were performed using the SPSS software (SPSS Standard version 23.0, SPSS Inc., Chicago, IL). Continuous variables were presented as means ± SD, minimum value, and maximum value. Categorical variables were classified and shown as numbers and percentages. Differences between groups were tested by Student's *t*-test, chi-square test, or rank-sum test, respectively. Significant differences were defined as *P* < 0.05.

## 3. Results

### 3.1. Basic Characteristics

Diseases were classified using ICD-10. Of the 95 included diseases, diseases of the genitourinary system accounted for the largest proportion (*n* = 14, 14.74%); other classifications proportional from high to low in turn were diseases of the nervous system (*n* = 12, 12.63%), diseases of the digestive system (*n* = 10, 10.53%), diseases of the respiratory system (*n* = 8, 8.42%), neoplasms (*n* = 8, 8.42%), certain infectious and parasitic diseases (*n* = 7, 7.37%), diseases of the musculoskeletal system and connective tissue (*n* = 7, 7.37%), diseases of the skin and subcutaneous tissue (*n* = 7, 7.37%), diseases of the blood and blood-forming organs and certain disorders involving the immune mechanism (*n* = 7, 7.37%), diseases of the circulatory system (*n* = 5, 5.26%), diseases of the eye and adnexa (*n* = 4, 4.21%), mental and behavioral disorders (*n* = 3, 3.16%), endocrine, nutritional, and metabolic diseases (*n* = 2, 2.11%), and diseases of the ear and mastoid process (*n* = 1, 1.05%). The 95 dominant diseases covered almost all disease systems.

Although there was specific TCM therapy for each disease, not every one of them had a TCM disease code. The results showed that 33 (34.74%) of the 95 diseases had no TCM disease name and used a western medicine name in clinical practice.

Length of hospital stay ranged from ≤7 days to ≤35 days. As is shown in Table 1, a total of 50 (52.63%) diseases' average length of stay was ≤14 days and maximally not exceeding 35 days.

### 3.2. Application of TCM

The application of TCM was summarized in Table 2; Chinese herbal decoction pieces and Chinese patent drugs were all used in the 95 dominant diseases of TCM. However, the utilization of Chinese medical injections varied from 28.57 to 100.00%, with a total rate of 63.16%. The lowest rate (2/7) of Chinese medical injections use was seen in diseases of the skin and subcutaneous tissue.

### 3.3. Application of TCM External Treatment

Table 3 and Table 4 indicated that, for each of included diseases, there was at least one TCM external therapy, and the number of external therapies can reach a maximum of 10. Acupuncture, moxibustion, manipulation, and Chinese medical plastering therapy were most widely applied in these diseases. Among them, acupuncture included ear acupuncture, collateral pricking, cutaneous needle, plum-blossom needle, and many other techniques. Uncommon characteristic therapies of TCM such as acupoint injection, TCM ion introduction, TCM enema, and TCM positive ridge were also widely used in these diseases.

## 4. Discussion

Our study found that the 95 TCM dominant diseases covered multiple systems, mainly the genitourinary, nervous, and digestive systems. However, the diseases' code of TCM was incomplete and remained to be revised and improved. The length of hospital stay was mainly ≤14 days. Each disease has its own Chinese herbal decoction pieces and Chinese patent drugs. Although therapeutically effective [13–15], Chinese medical injections have not been widely used, which may be because of the controversy on their safety [16]. For the 95 TCM dominant diseases, there were many alternative external treatments of TCM. Therapies such as acupuncture and moxibustion have been widely recognized for their efficacy, easy operation, and low cost and played an important role in the therapy process of many diseases [17–19].

For thousands of years, TCM has been widely used in clinical practice in China. How to inherit and develop the advantages of TCM in the diagnosis and treatment of diseases and health maintenance is still a hot topic [20]. Some scholars have proposed that strategy should, with clinical efficacy at the core, be developed based on a single disease. A study conducted in a TCM hospital indicated that, in health economics, the TCM dominant diseases are characterized by difficulties in treatment, a longer length of hospital stay, and higher hospitalization costs [21]. But evidence from other research suggested that because of the long-term therapeutic effect of TCM, the number of readmissions and total expenses of treatment reduced with the participant of Chinese medical treatment [22]. For example, in the TCM treatment of acute myocardial infarction, the readmission rate due to angina during the 6-month follow-up in the treatment group (2.96%) was significantly lower than that in the control group (7.88%) [23]. Therefore, TCM dominant diseases are ubiquitous and need us to excavate through research.

The evaluation criterion of TCM dominant diseases exactly follows the principle of focusing on a single disease and with clinical efficacy at the core. Under the guidelines of these evaluation criteria, the potential TCM dominant diseases can be evaluated one by one, and the scope of TCM dominant diseases can be continuously expanded and enriched according to the criteria of the evidence grade of evidence-based medicine. Currently, the level of evidence from TCM trials is generally low [24]. Moreover, a large number of diseases were considered TCM dominant diseases by experts but lacked high-quality evidence. Therefore, it is important to establish mature evaluation criteria for TCM dominant diseases as soon as possible. With the guidance of evaluation criteria of TCM dominant diseases, finding the direction of the topic of high-quality original clinical research will also be easier [25, 26].

However, the concept of TCM dominant diseases has been put forward for decades and a large number of clinical trials have also demonstrated the superiority of TCM in the treatment process of some diseases. There have been no clear regulations to elucidate which diseases belong to the dominant diseases of TCM until the list of dominant diseases of TCM issued by the Chinese State Administration of Traditional Chinese Medicine in 2019, which systematically summarized the dominant diseases of TCM on a national scale for the first time and described their diagnosis and treatment protocols and clinical pathways in detail, providing important references for clinical practice. As the list is derived from the collective views of experts, there is a level of subjectivity in the process of developing the list.

Future studies could start with diseases in which TCM was widely used with clear therapeutic effect and an accepted TCM treatment to unearth more TCM dominant diseases. On the other hand, high-quality original research is also warranted to reinforce its theoretical basis.

## 5. Conclusion

For all the 95 TCM dominant diseases, there were definite TCM treatment protocols, clinical pathways, length of hospital stay, specific Chinese herbal decoction pieces, and Chinese patent drugs. Various characteristic TCM external therapies were widely applied in these diseases. This study may offer some reference for the establishment of the evaluation criterion of TCM dominant diseases.

## Figures and Tables

**Table 1:** Basic characteristics of 95 dominant diseases of traditional Chinese medicine.

Disease classification	Diseases		Diseases' coding of TCM		Length of hospital stay				
	N	Proportion (%)	Available	No	≤7	≤14	≤21	≤28	≤35
Diseases of the genitourinary system	14	14.74	12	2	0	14	0	0	0
Diseases of the nervous system	12	12.63	12	0	0	3	4	5	0
Diseases of the digestive system	10	10.53	9	1	1	2	4	3	0
Diseases of the respiratory system	8	8.42	7	1	1	6	0	1	0
Neoplasms	8	8.42	3	5	0	5	1	1	1
Certain infectious and parasitic diseases	7	7.37	1	6	0	4	2	1	0
Diseases of the musculoskeletal system and connective tissue	7	7.37	3	4	0	2	3	2	0
Diseases of the skin and subcutaneous tissue	7	7.37	4	3	1	1	2	3	0
Diseases of the blood and blood-forming organs and certain disorders involving the immune mechanism	7	7.37	0	7	0	5	2	0	0
Diseases of the circulatory system	5	5.26	3	2	0	4	1	0	0
Diseases of the eye and adnexa	4	4.21	3	1	0	0	1	3	0
Mental and behavioral disorders	3	3.16	3	0	1	2	0	0	0
Endocrine, nutritional, and metabolic diseases	2	2.11	1	1	0	2	0	0	0
Diseases of the ear and mastoid process	1	1.05	1	0	1	0	0	0	0
Total	95	100	62	33	5	50	20	19	1

TCM, traditional Chinese medicine.

**Table 2:** Application of TCM in the treatment of 95 dominant diseases of TCM.

Disease classification	Number of diseases	Chinese herbal decoction pieces		Chinese patent drugs		Chinese medical injections	
		*n*	Proportion (%)	*n*	Proportion (%)	*n*	Proportion (%)
Diseases of the genitourinary system	14	14	100.00	14	100.00	6	42.86
Diseases of the nervous system	12	12	100.00	12	100.00	8	66.67
Diseases of the digestive system	10	10	100.00	10	100.00	7	70.00
Diseases of the respiratory system	8	8	100.00	8	100.00	5	62.50
Neoplasms	8	8	100.00	8	100.00	7	87.50
Certain infectious and parasitic diseases	7	7	100.00	7	100.00	7	100.00
Diseases of the musculoskeletal system and connective tissue	7	7	100.00	7	100.00	5	71.43
Diseases of the skin and subcutaneous tissue	7	7	100.00	7	100.00	2	28.57
Diseases of the blood and blood-forming organs and certain disorders involving the immune mechanism	7	7	100.00	7	100.00	5	71.43
Diseases of the circulatory system	5	5	100.00	5	100.00	2	40.00
Diseases of the eye and adnexa	4	4	100.00	4	100.00	3	75.00
Mental and behavioral disorders	3	3	100.00	3	100.00	1	33.33
Endocrine, nutritional, and metabolic diseases	2	2	100.00	2	100.00	1	50.00
Diseases of the ear and mastoid process	1	1	100.00	1	100.00	1	100.00
Total	95	95	100.00	95	100.00	60	63.16

**Table 3:** Application of TCM external treatment in 95 dominant diseases of TCM.

Disease classification	Number of diseases	Number of optional TCM external therapies	Number of optional TCM external therapies/number of diseases
Diseases of the musculoskeletal system and connective tissue	7	47	6.71
Diseases of the skin and subcutaneous tissue	7	32	4.57
Diseases of the circulatory system	5	22	4.40
Diseases of the respiratory system	8	34	4.25
Diseases of the ear and mastoid process	1	4	4.00
Diseases of the nervous system	12	46	3.83
Neoplasms	9	34	3.78
Diseases of the genitourinary system	14	47	3.36
Diseases of the blood and blood-forming organs and certain disorders involving the immune mechanism	6	19	3.17
Diseases of the digestive system	10	29	2.90
Diseases of the eye and adnexa	4	11	2.75
Certain infectious and parasitic diseases	7	18	2.57
Endocrine, nutritional, and metabolic diseases	2	5	2.50
Mental and behavioral disorders	3	6	2.00
Total	95	354	3.73

**Table 4:** Application of TCM external treatment in 95 dominant diseases of TCM (detailed).

Serial number	Disease name in western medicine	Disease code in ICD 10	Disease code in ICD 11	Optional TCM external therapies	Disease classification
1	Viral encephalitis (acute stage)	A86/*G*05.1	1C80	(1) Acupuncture ① Ear acupuncture ② Collateral pricking ③ Cutaneous needle ④ Plum-Blossom needle	Certain infectious and parasitic diseases
2	Dengue fever	AP0 × 00	1D2Z	(1) TCM external washing (2) TCM enema	Certain infectious and parasitic diseases
3	Ramsay Hunt syndrome	B02.203	8B88.Y	(1) Acupuncture ① Body acupuncture ② Electroacupuncture (2) Moxibustion (3) Cupping (4) Manipulation	Certain infectious and parasitic diseases
4	Hand, foot, and mouth disease（severe ）	B08.401	1F05.0	(1) Acupuncture (2) Manipulation	Certain infectious and parasitic diseases
5	Hepatitis B virus associated glomerulonephritis	B10.910+	GB40 and1E51.0Z	(1) Acupuncture (2) Electronic biofeedback therapeutic instrument (3) TCM enema	Certain infectious and parasitic diseases
6	Viral hepatitis E	B17.202	1E51.3	(1) Acupuncture (2) Ear pressure beans (3) TCM enema (4) Moxibustion	Certain infectious and parasitic diseases
7	Infectious mononucleosis (without serious complications)	B27.901	1D81.Z	(1) TCM spray pharynx (2) TCM compress	Certain infectious and parasitic diseases
8	Malignant neoplasm of breast (perioperative period)	C50.900	2C6Z	(1) Acupuncture (2) Acupoint application (3) Moxibustion (4) TCM hot compress	Neoplasms
9	Malignant neoplasm of breast (consolidation stage)	C50.902	2C6Z	(1) Acupuncture (2) Moxibustion (3) Ear pressure beans (4) TCM diagnosis and treatment equipment	Neoplasms
10	Malignant neoplasm of ovary	C56.X00	2C73.Z	(1) TCM application (2) Acupuncture (3) Ear pressure beans (4) Cupping (5) Moxibustion	Neoplasms
11	Malignant neoplasm of prostate	C61.x00	2C82.Z	(1) TCM soaking (2) Moxibustion (3) Acupoint application (4) Acupuncture	Neoplasms
12	Malignant lymphoma/aggressive lymphoma (after chemotherapy)	C82	2B33.5	(1) TCM compress (2) Acupuncture; (3) Moxibustion	Neoplasms
13	Acute lymphoblastic leukemia	C91.001	2B33.3	(1) Acupoint application (2) Ear pressure beans (3) TCM soaking (4) Medicated diet and dietotherapy	Neoplasms
14	Acute myeloblastic leukemia (elderly)	C92.004	2A60.3Z	(1) Ear pressure beans (2) Moxibustion (3) Acupoint application (4) Acupoint ironing	Neoplasms
15	Acute promyelocytic leukemia (low and intermediate risk)	C92.401，M986604/3	2A60.0	(1) TCM compress	Neoplasms
16	Polycythemia vera	D45.X01	2A20.4	(1) TCM foot bath (2) Acupoint application (3) Acupuncture (4) TCM compress (5) Bloodletting therapy	Neoplasms
17	Megaloblastic anemia	D53.100	3A01.Y	(1) Medicated diet and dietotherapy (2) Acupuncture (3) Moxibustion	Diseases of the blood and blood-forming organs and certain disorders involving the immune mechanism
18	Purpura nephritis (children)	D69.005	GB55.Y/3B60	(1) Moxibustion (2) Ear pressure beans (3) Low-frequency pulse electrical stimulation (4) TCM fumigation	Diseases of the blood and blood-forming organs and certain disorders involving the immune mechanism
19	Secondary thrombocytopenia (after chemotherapy)	D69.602	3B64.1Y	(1) TCM compress (2) Acupoint application	Diseases of the blood and blood-forming organs and certain disorders involving the immune mechanism
20	Leukopenia(after chemotherapy)	D72.901	4B00.01	(1) Acupuncture (2) Moxibustion (3) Acupoint injection	Diseases of the blood and blood-forming organs and certain disorders involving the immune mechanism
21	Essential thrombocythaemia	D47.300	3B63.1Z	(1) Acupuncture (2) Moxibustion (3) Manipulation (4) TCM compress	Diseases of the blood and blood-forming organs and certain disorders involving the immune mechanism
22	Anemia (tumor associated)	D52.100	3A71.0	(1) Moxibustion (2) Acupoint application (3) Medicated diet and dietotherapy	Diseases of the blood and blood-forming organs and certain disorders involving the immune mechanism
23	Abnormality of lipid metabolism (diabetic)	E14.600	5C62and5A14	(1) Acupuncture (2) Moxibustion (3) Ear acupuncture (4) Manipulation	Endocrine, nutritional and metabolic diseases
24	Diabetic foot	E14.606	BD54	(1) TCM compress	Endocrine, nutritional and metabolic diseases
25	Mental and behavioral disorders due to the use of alcohol	F10.900	6C40.6Z	(1) Transcutaneous electrical acupoint stimulation (2) Ear acupuncture (3) Bloodletting therapy	Mental and behavioral disorders
26	Acute stress response	F43.0	QE84	(1) Acupuncture	Mental and behavioral disorders
27	Dissociative [conversion] disorders	F44	6B60.Z	(1) Acupuncture (2) Acupoint application	Mental and behavioral disorders
28	Motor neuron disease	G12.210	8B60.Z	(1) Acupuncture (2) Moxibustion (3) Acupoint injection (4) Cutaneous needle (5) Manipulation	Diseases of the nervous system
29	Parkinsonism-plus syndrome	G20.02	8A00.Y	(1) Acupuncture: ① scalp acupuncture; ② body acupuncture (2) TCM soaking (3) Moxibustion (4) Manipulation	Diseases of the nervous system
30	Parkinson disease (with bladder dysfunction)	G20.02	8A00.Y	(1) Acupuncture (2) Moxibustion (3) TCM compress (4) TCM psychotherapy (5) Low-frequency pulse electrical stimulation	Diseases of the nervous system
31	Alzheimer disease	G30.9	8A20	(1) Sensory irritation (2) Cognitive stimulation (3) Emotional intervention	Diseases of the nervous system
32	Neuromyelitis optica	G36.001	8A43.Z	(1) Acupuncture	Diseases of the nervous system
33	Cervical headache	G44.801	8A84.Y	(1) Acupuncture (2) Manipulation (3) Traction treatment (4) Moxibustion	Diseases of the nervous system
34	Posterior circulation ischemia	G45.0	8B10.Y	(1) TCM compress (2) Acupuncture	Diseases of the nervous system
35	Carpal tunnel syndrome	G56.001	8C10.0	(1) Manipulation (2) Electroacupuncture (3) TCM hot compress (4) TCM soaking	Diseases of the nervous system
36	Ankle canal syndrome	G57.502	8C1Z	(1) Manipulation (2) Acupuncture (3) Electroacupuncture (4) TCM hot compress (5) TCM soaking; 6)Moxibustion	Diseases of the nervous system
37	Chronic inflammatory demyelinating polyneuropathy	G61.801	8C01.3	(1) Acupuncture (2) Moxibustion (3) Manipulation (4) TCM soaking	Diseases of the nervous system
38	Myasthenia gravis	G70.000	8C60.Z	(1) Acupoint injection (2) Cutaneous needle (3) TCM soaking (4) Manipulation (5) Acupoint application	Diseases of the nervous system
39	Muscular dystrophy (progressive)	G71.001	8C70	(1) External TCM (2) Acupoint injection (3) TCM enema	Diseases of the nervous system
40	Retinal artery occlusion (branch)	H34.202	9B74.0	(1) Acupuncture (2) Moxibustion (3) Ear pressure beans (4) Acupoint injection	Diseases of the eye and adnexa
41	Senile macular degeneration (atrophic) (exudative)	H35.311	9B75.0Y	(1) Acupuncture (2) Moxibustion	Diseases of the eye and adnexa
42	Vitreous hemorrhage	H43.100	9B83	(1) Acupoint injection (2) Ocular iontophoresis (3) Acupuncture (4) Moxibustion	Diseases of the eye and adnexa
43	External ophthalmoplegia	H49.807	9C82.Z	(1) Acupuncture	Diseases of the eye and adnexa
44	Ménière's disease	H81.000	AB31.0	(1) Acupuncture: ① body acupuncture; ② ear acupuncture; ③ scalp acupuncture (2) Moxibustion (3) Acupoint injection (4) Ear pressure beans	Diseases of the ear and mastoid process
45	Viral myocarditis (children)	I40.001\I41.1	BC42.1	(1) Acupuncture (2) Manipulation (3) Acupoint application (4) Acupoint injection	Diseases of the circulatory system
46	Diabetic peripheral angiopathy	I79.202	BD53.Y	(1) Acupuncture (2) Moxibustion (3) TCM fumigation	Diseases of the circulatory system
47	Thrombophlebitis	I80.902	BD70.Z	(1) TCM compress	Diseases of the circulatory system
48	Varicocele	I86.101	5A81.1	(1) Acupuncture (2) Moxibustion (3) Needle-picking (4) Acupoint application (5) Acupoint injection	Diseases of the circulatory system
49	Mesenteric lymphadenitis (children)	I88.002	BD90.1	(1) Acupoint application (2) Manipulation (3) Moxibustion (4) TCM ion introduction (5) TCM hot iron (6) TCM soaking (7) Acupuncture (8) Ear pressure beans (9) Cupping	Diseases of the circulatory system
50	Acute tonsillitis (children)	J03.900	CA03.Z	(1) Acupoint application (2) Acupuncture (3) Moxibustion	Diseases of the respiratory system
51	Mycoplasma pneumonia	J15.702	CA40.04	(1) TCM chest compress (2) Acupoint application (3) Cupping (4) TCM ion introduction (5) Umbilical therapy	Diseases of the respiratory system
52	Severe community-acquired pneumonia	J15.903	CA40.Z	(1) TCM ion introduction (2) TCM enema	Diseases of the respiratory system
53	Hospital-acquired pneumonia	J18.8	CA40.Z	(1) Acupuncture (2) TCM atomization inhalation (3) TCM enema (4) TCM compress (5) Skin scraping therapy	Diseases of the respiratory system
54	Acute tracheitis/bronchitis	J20.902	CA42.Z	(1) Acupoint application (2) Moxibustion (3) Acupuncture (4) Cupping (5) Stone needle therapy	Diseases of the respiratory system
55	Bronchiolitis	J21.902	CA40.Z	(1) Infantile tuina (2) TCM ion introduction (3) Acupoint application (4) TCM chest compress (5) TCM enema (6) Acupuncture (7) Ear pressure beans (8) Chiropractic therapy	Diseases of the respiratory system
56	Pharyngeal abscess	J36.X00; J39.001; J39.003; J05.100	CA0K.0	(1) Acupuncture: ① body acupuncture; ② Bloodletting therapy (2) TCM external therapy: ① Insufflating medicinal powder, gargle, dissolving in the mouth, nebulization, compress, and evacuation of pus (3) Lifting and scraping therapy	Diseases of the respiratory system
57	Bronchiectasis	J47.x00	CA24	(1) Acupuncture (2) Moxibustion (3) Acupoint application (4) Acupoint injection	Diseases of the respiratory system
58	Gastritis (*Helicobacter pylori*-associated) (refractory)	A49809 + （……）^*∗*^	DA42.1	(1) Acupuncture (2) Moxibustion (3) Abdominal paste massage (4) Acupoint application	Diseases of the digestive system
59	Cryptitis(anal)	K62.801	DB70.Z	(1) TCM fumigation (2) TCM compress (3) Turunda	Diseases of the digestive system
60	Hypertrophy of anal papilla	K62.806	DB71.2	(1) TCM fumigation (2) Turunda (3) TCM enema	Diseases of the digestive system
61	Alcoholic cirrhosis of liver	K70.301	DB94.2	(1) Acupoint application	Diseases of the digestive system
62	Hepatic failure (hepatitis B related) (early stage)	K72.004	DB99.7and1E51.0Z	(1) TCM enema (2) TCM rectal instillation	Diseases of the digestive system
63	Chronic hepatic failure	K72.101	DB99.8	(1) TCM enema (2) TCM compress	Diseases of the digestive system
64	Ascites (hepatitis B related) (hepatic sclerosis)	K74 ＋ R18	1E51.0Z/DB93.1 + ME04.0	(1) TCM umbilical therapy (2) Acupuncture (3) TCM enema	Diseases of the digestive system
65	Cholestatic hepatitis	K75.802	DB97.Y	(1) TCM enema (2) Liver disease therapeutic apparatus (3) Acupuncture (4) Moxibustion	Diseases of the digestive system
66	Gallstone	K80.203	DC11	(1) Acupuncture (2) Moxibustion (3) Ear pressure beans (4) TCM enema (5) TCM application	Diseases of the digestive system
67	Cholangitis (primary) (sclerosing)	K83.0	DB96.2Z	(1) TCM fumigation (2) Liver disease therapeutic apparatus	Diseases of the digestive system
68	Impetigo	L01.000	1B72.Z	(1) TCM external therapy (2) Acupuncture (3) Moxibustion	Diseases of the skin and subcutaneous tissue
69	Pilonidal cyst (sacrococcygeal)	L05.900	EG63.0	(1) TCM compress (2) TCM fumigation	Diseases of the skin and subcutaneous tissue
70	Pustular psoriasis	L40.100	EA90.4	(1) Acupuncture (2) Triangular needle quick puncture (3) Cupping and exsanguination	Diseases of the skin and subcutaneous tissue
71	Pemphigus	L10	EB40.Z	(1) TCM collapse stains (2) TCM scrub treatment (3) Moxibustion (4) TCM bath (5) Acupoint injection (6) Acupuncture	Diseases of the skin and subcutaneous tissue
72	Erythroderma psoriasis	L40.801	EA90.3	(1) TCM wet compress (2) TCM bath (3) TCM ointment or oil (4) Acupoint application (5) Acupuncture (6) Moxibustion (7) Cupping	Diseases of the skin and subcutaneous tissue
73	Chronic actinic dermatitis	L57.801	EJ30.1	(1) TCM external therapy (2) Acupuncture (3) Moxibustion (4) Ear pressure beans	Diseases of the skin and subcutaneous tissue
74	Allergic cutaneous vasculitis	L95.802	4A44.BZ	(1) TCM collapse stains (2) TCM scrub treatment (3) Acupuncture (4) Moxibustion (5) Ear acupuncture (6) TCM hydronium spray (7) Acupoint application	Diseases of the skin and subcutaneous tissue
75	Lupus nephritis	M32.101+	4A40.0Y	(1) Acupuncture (2) Moxibustion	Diseases of the musculoskeletal system and connective tissue
76	Juvenile idiopathic scoliosis	M41.992	FA70.1	(1) Tendon-soothing manipulation (2) TCM hot compress (3) TCM fumigation (4) Acupuncture (5) Manipulation (6) Chiropractic treatment (7) Needle knife treatment (8) Positive ridge (9) Traction (10) Moxibustion	Diseases of the musculoskeletal system and connective tissue
77	Spondylolisthesis (lumbar)	M43.162	FA81.Z&XA0D60	(1) Tendon-soothing manipulation (2) TCM hot compress (3) TCM fumigation (4) Acupuncture (5) Manipulation (6) Needle knife treatment (7) Positive ridge (8) Traction (9) Moxibustion	Diseases of the musculoskeletal system and connective tissue
78	Contracture of muscle (gluteal)	M62.405	FB32.4&XA48F2	(1) Manipulation (2) Acupuncture (3) Moxibustion (4) TCM hot compress (5) TCM soaking	Diseases of the musculoskeletal system and connective tissue
79	Metatarsalgia	M77.401	FB54.4	(1) Body acupuncture (2) Ear acupuncture (3) Acupoint application (4) Moxibustion (5) TCM hot compress	Diseases of the musculoskeletal system and connective tissue
80	Fibromyalgia	M79.792	MG30.01	(1) TCM health exercises (2) Acupoint application (3) Acupuncture (4) TCM bath (5) TCM fumigation (6) TCM ion introduction (7) Musical therapy (8) Moxibustion	Diseases of the musculoskeletal system and connective tissue
81	Degenerative lumbar spinal stenosis	M48.061	FA82	(1) Tendon-soothing manipulation (2) TCM hot compress (3) Acupuncture (4) Manipulation (5) Needle knife treatment (6) Positive ridge (7) Traction (8) Moxibustion	Diseases of the musculoskeletal system and connective tissue
82	Acute glomerulonephritis	N00 + B95.5	GB40	(1) Acupuncture: ① body acupuncture ② Ear acupuncture	Diseases of the genitourinary system
83	Primary nephrotic syndrome (primary) (children)	N04.900	GB41	(1) Moxibustion (2) Acupuncture (3) TCM compress	Diseases of the genitourinary system
84	Idiopathic membranous nephropathy	N05.201	GB41	(1) Medicated diet and dietotherapy (2) TCM soaking (3) Acupoint application	Diseases of the genitourinary system
85	Acute pyelonephritis	N10.X01	GB51	(1) Acupuncture	Diseases of the genitourinary system
86	Urolithiasis	N20.951	GB70.Z	(1) Acupuncture (2) Moxibustion	Diseases of the genitourinary system
87	Hyperplasia of prostate (benign)	N40	GA90	(1) Acupuncture (2) TCM umbilical therapy (3) TCM enema (4) TCM enema	Diseases of the genitourinary system
88	Orchitis/epididymitis (acute/chronic)	N45.903; N45.902	GB02.Y	(1) TCM external therapy (2) Acupuncture (3) Moxibustion	Diseases of the genitourinary system
89	Vesiculitis (seminal)	N49.001	GB07.0	(1) TCM enema (2) Acupuncture (3) Moxibustion	Diseases of the genitourinary system
90	Mastitis (plasma cell)	N61.X02	GB20.0	(1) TCM application (2) Acupoint application (3) TCM ion introduction	Diseases of the genitourinary system
91	Granulomatous lobular mastitis (abscess)	N61.x07	GB21.Y	(1) TCM compress (2) Ironing therapy (3) TCM external Washing/TCM fumigation (4) Moxibustion (5) Collateral prickingcupping (6) TCM ion introduction (7) Catheter perfusion (8) TCM external therapy	Diseases of the genitourinary system
92	Pelvic congestion syndrome	N94.803	GA34.Y	(1) Rectal administration (2) Ironing therapy (3) TCM compress (4) Acupuncture (5) Moxibustion	Diseases of the genitourinary system
93	Minimal change nephropathy (adult)	NO5.004	GB40	(1) TCM soaking (2) Moxibustion (3) T CM fumigation	Diseases of the genitourinary system
94	Hyperemesis gravidarum	Q21.951	JA60.Z	(1) Acupuncture (2) Moxibustion (3) Cupping (4) Ear pressure beans	Diseases of the genitourinary system
95	Polyuria (neurogenic)	R35.X51	MF50.0	(1) Acupuncture (2) Ear pressure beans (3) Acupoint application (4) Manipulation	Diseases of the genitourinary system

## Data Availability

The datasets analyzed during the current study are available from the corresponding author on reasonable request.
